RETRACTED

# Image Matching Algorithm Based on the Pattern Recognition Genetic Algorithm

**DOI:** 10.1155/2022/7760437

**Published:** 2022-03-09

**Authors:** Lipeng Si, Xiuhua Hu, Baolong Liu

**Affiliations:** School of Computer Science and Engineering, Xi'an Technological University, Xi'an 710021, Shaanxi, China

## Abstract

Image matching is an important topic in image processing. Matching technology plays an important role in and is the basis for image understanding. In order to solve the shortcomings of slow image matching and low matching accuracy, a matching method based on improved genetic algorithm is proposed. The main improvement of the algorithm is the use of self-identifying crossover operators for crossover operations to avoid premature population maturity. According to the characteristics of the image data, new intersection and mutation operators are defined by the new coding method. The sampling method is used to initialize the population method, introduce an evolution strategy, reduce the number of iterations, and effectively reduce the amount of calculation. The experimental results show that the algorithm can guarantee the matching accuracy and that the calculation time is much shorter than that of the original algorithm. In addition, the image matching calculation time per frame of the algorithm is basically unchanged, which is convenient for engineering applications.

## 1. Introduction

Image matching is an important subject in image processing. It has broad application prospects in computer vision, moving target tracking and recognition, motion compensation in sequence image compression, and medical image processing. Matching technology plays an important role in understanding images.

Image correlation matching tracking techniques are the basic means by which optoelectronic imaging systems track moving and stationary surfaces. For close-range targets or large-size surface targets, the target image occupies most of the field of view or fills the field of view, and the amount of data and image-related matching is computationally large [1]. Image matching technology has become more and more prominent in the field of image processing. It has been widely used in many fields and has high research value and application value [2, 3]. With the rapid development of integrated circuit (IC) technology and microelectronics technology, the integration and performance of field programmable gate arrays (FPGA) have been greatly improved. Using the super parallel processing capabilities of FPGAs, some image matching algorithms can be used [4, 5]. Hardware implementation can greatly accelerate the speed of matching.

The SSDA algorithm can guarantee the global optimality of image matching, but the SSDA algorithm can only adopt the MAD matching criterion and cannot adopt the NPROD matching criterion. Furthermore, according to the target position, the matching time required for each frame of image is uncertain, which is not convenient for engineering implementation [6–9]. The MPSA algorithm can use the MAD and NPROD matching criteria, and the matching time required for each frame of image is substantially constant. However, there may be a mismatch in the MPSA algorithm, especially in the case of low contrast. It is exchanged for the loss of matching accuracy [10]. Therefore, under the premise of ensuring the best matching accuracy, the computational complexity of image correlation matching is greatly reduced.

RETRACTED

The amount of computation for image correlation matching depends on the search strategy it uses to find the best match location. Existing methods use a traversal search strategy, so the reduction in computation is limited. It is difficult to achieve a substantial breakthrough in reducing calculations [11–15]. This is a common shortcoming of existing image correlation matching algorithms. Genetic algorithm is a new theory and new method developed in recent years. It uses a non-traversal search strategy to ensure that the search results have global optimality, and the amount of computation required is much smaller than the traversal search [16–18]. The traditional image matching method's search strategy is to search all points on the area, so its efficiency is very low. This means that a lot of search time will be wasted on non-target points, which is not what we want. Therefore, improving the search strategy is of great significance to improve the matching efficiency. On this basis, the application of genetic algorithm in image matching came into being. At present, genetic algorithms have been widely used in image restoration, image feature extraction, image calibration, image segmentation, image recognition, image compression, and image retrieval [19]. Since the genetic algorithm is a random search algorithm, it starts searching from multiple points instead of one. This makes it possible to find the non-ergodicity of the overall optimal solution genetic algorithm with a large probability and to ensure the robustness of the search efficiency genetic algorithm, making it less susceptible to image noise [20, 21].

In this paper, the genetic algorithm is applied to the research of image correlation matching algorithm, and a fast image correlation matching algorithm is proposed. Combined with the characteristics of image matching itself, a new coding method is used to define new intersection and mutation operators. The calculation amount is effectively reduced, the matching precision is greatly improved, and good experimental results are obtained. Under the same matching effect, the algorithm is more than 100 times faster in calculation speed than the original algorithm. The NPROD matching criterion is used to improve the matching accuracy under low SNR conditions. The algorithm also has the advantage that the image matching calculation time per frame is basically constant, which is convenient for use in practical systems.

RETRACTED

## 2. Proposed Method

### 2.1. Pattern Recognition

Pattern recognition is the use of mathematical techniques to study the automatic processing and interpretation of patterns. We refer to the environment and the object as “models.” With the development of computer technology, human beings are likely to study complex information processing processes. An important form of information processing is through biometric environments and objects. Of particular importance to humans is the identification of optical information (obtained through visual organs) and acoustic information (obtained through auditory organs). These are two important aspects of pattern recognition. Representative products available on the market include optical character recognition and speech recognition systems.

When people observe things or phenomena, they often look for differences between them and other things or phenomena, and for each purpose, constitute each similar or different things or phenomena. Character recognition is a typical example. For example, the number “4” can be written in a variety of ways, but all belong to the same category. More importantly, even if you do not see the “4” of a certain method before, you can classify it as the category to which “4” belongs. This ability of thinking in the human brain constitutes the concept of a “model.” In the above example, as long as you know a limited number of things or phenomena in this collection, the concepts of patterns and collections are separate and you can identify many things or phenomena that belong to the collection. To emphasize the inference of the totality of things or phenomena from certain individual things or phenomena, we refer to these individual things or phenomena as patterns. Some scholars believe that the whole category should be called a model. A specific object, such as the Great Hall of the People, is called a sample in the “house” model. The different meanings of this noun are easily clarified from the context. Pattern recognition is the basic wisdom of human beings. With the advent of computers in the 1940s and the rise of artificial intelligence in the 1950s, people certainly wanted to use computers to replace or extend part of the human brain. (Computer) pattern recognition developed rapidly and became a new discipline in the early 1960s. Pattern recognition refers to the processing and analysis of various forms (digital, textual, and logical) of information that characterize things or phenomena. The process of describing, identifying, classifying, and interpreting things or phenomena is an important part of information science and artificial intelligence. Pattern recognition research focuses on two aspects. The first is the research content of physiologists, psychologists, biologists, and neurophysiologists. The second is how to use a computer to implement pattern recognition theory and methods for a given task. Systematic research results have been achieved. A computer application identifies and classifies a set of events or processes. These objects are different from the information in digital form and are called pattern information.

RETRACTED

The number of categories classified by pattern recognition is determined by a particular identification problem. Sometimes, the actual number of categories cannot be known at the beginning, and the system must be identified after repeatedly observing the identified objects. Pattern recognition is related to statistics, psychology, linguistics, computer science, biology, and cybernetics. It has a cross-relationship with the research of artificial intelligence and image processing. For example, adaptive or ad hoc pattern recognition systems include artificial intelligence learning mechanisms; landscape understanding and natural language understanding of artificial intelligence research also include pattern recognition issues. Another example is the technique of applying image processing in the preprocessing and feature extraction steps in pattern recognition; image analysis in image processing also applies pattern recognition techniques.

### 2.2. Genetic Algorithm

Since the Netherlands proposed genetic algorithms, they have been extensively studied in academia. Genetic algorithms have many different forms of improvement for different applications. Genetic algorithms have also been applied to imaging tracking. 1. The effect of the initial population on the algorithm search speed: genetic algorithms are limited by the computational power of the actual system. It directly affects the optimization speed and search effect of the algorithm. The initial population (first generation population) is usually obtained by uniform sowing or random seeding. If the genetic score of the initial population is high, the greater the probability of containing the effective gene, the higher the convergence speed of the algorithm. The initial population is obtained by a uniform seeding method; that is, *N* (*N* is a population size) seed is obtained as a first generation population at equal intervals in the search domain. After the first *M* genetic iteration, the algorithm searches for the vicinity of each local maximum and then *N* genetic iterations to converge to global optimality. If a valid initialization method is used, the initial population itself can be concentrated near each local maximum (assuming a global maximum is found). Obviously, in order to converge to the same result, a genetic algorithm using an efficient initialization method requires fewer genetic iterations than a uniform seeding method, so the search speed is fast. For the specific application of image correlation matching, the initial population selection of genetic algorithm mainly has the following methods. (1) An initialization method for specifying a probability distribution. That is to say, the distribution of the initial population in the entire search domain conforms to a specific probability distribution. For a particular application environment, a specific probability distribution can be specified to obtain an initial population. For example, in imaging tracking applications, depending on the continuity characteristics of the target motion, the target position in the current frame image being not far from the target position detected by the previous frame image is a high probability event. Therefore, when processing the current frame image, the number of seeds to be planted near the target position of the previous frame should also be large. (2) Drop resolution preferred method: a matching surface of the low resolution image of the target image and the original image is calculated, and the first *N* point positions having the largest matching degree are selected as the initial population. The statistics show that the autocorrelation length of the general image (the amount of displacement when the autocorrelation coefficient drops to 1e = 0.368) is about 20 pixels. Therefore, the correlation surface calculated after the resolution is lowered has a high similarity to the original correlation surface, thereby ensuring the effectiveness of the initialization method. (3) The method of reducing the dimension. Low dimensional similarity is a necessary condition for high dimensional similarity.

RETRACTED

As mentioned above, the initial population has a higher genetic score and a high probability of containing a valid gene, so the initial population distribution is near each local maximum. In the choice of the initial population, we must follow this standard. In the various initialization methods described above, the optimal solution obtained by initialization is not necessarily the local optimal solution of the system (the former is a necessary condition of the latter rather than a sufficient condition). Therefore, no matter which method is used, there is no guarantee that the seeding position must be close to the local optimum. When the seeding is far away from the local optimum area, the initialization effect is not as good as the uniform seeding effect, plus the calculation amount, the number of iterations is insufficient, and the population does not converge or only converges to the local optimum. Therefore, this paper proposes an effective genetic algorithm initialization strategy—a comprehensive strategy for controlling various initial methods of population spacing. The basic idea is to form a set of total *M* x *N* seed points (*N* is the population size) obtained by the *M* initialization method. Calculate and classify the matching degree of each point, and under the supervision of strictly controlling the population spacing, select the top *N* seed points with large matching degree as the initial population. The strategy can take advantage of each initialization method, so that the initial population falls near each local optimal region with a high probability, thereby greatly improving the search speed of the genetic algorithm. Optimization of crossover and mutation operators is as follows: genetic algorithms are implemented through a series of genetic operations. Common operations (or operators) include copy operations, cross operators, mutation operators, and selection operations. Among them, the properties of crossover operator and mutation operator reflect the search principle and search strategy of genetic algorithm. The mechanism of the crossover operator is equivalent to the inheritance in the biological sense, characterized by the production of individuals having a combination of genes similar to the father, which is mathematically represented as a converging operation. Under the condition of no mutation operation, the initial population undergoes *n* cross-genetic operations. When *n* is large enough, the population will eventually converge to local optimum. The so-called local optimum here is due to the convergence characteristics of the crossover operator, and it is impossible to generate an individual that is greatly different from the parent gene in the sense of probability. Therefore, as population algebra increases, the scope of search is limited and reduced. The mechanism of the mutation operator is exactly the opposite of the crossover operator, which is equivalent to a genetic mutation in the biological sense, which is characterized by the production of individuals having a combination of genes different from the father. It is expressed as a divergent operation in mathematics.

RETRACTED

Parameters in genetic algorithms, such as population, evolutionary algebra, crossover probability, and probability of mutation operation, affect the convergence speed of the algorithm and the global optimality of the result. However, it is difficult to accurately analyze the relationship between them by analytical methods. Appropriate parameter values are determined experimentally.

### 2.3. Fast Image Matching Based on the Genetic Algorithm

The purpose of image correlation matching is to find the best matching position of the template whose coordinates are the optimal solution of image correlation matching. Therefore, the most simple coding method is to directly use the binary code corresponding to the coordinates as the gene string. The significant difference between the binary codes corresponding to 127 and 128 in the code shape has an adverse effect on the convergence and matching accuracy of the algorithm. Select the gray-code coding scheme. Meet the requirements of similar spatial code neighbor code patterns.

The genetic algorithm used in this article is a multiobjective optimization genetic algorithm. Genetic algorithm is used for image correlation matching problem. The following six problems need to be solved: (1) coding; (2) initializing the population; (3) designing the fitness function; (4) designing the genetic operator; (5) introducing the competitive evolution strategy; (6) determining control parameters. In genetic algorithms, evolutionary processes are based on coding mechanisms. Holland's proposed genetic algorithm uses binary coding to represent an individual's genetic genotype. Therefore, the actual genetic genotype is a binary symbol string, which has the advantage of simple encoding and decoding operations, and can easily implement genetic operations such as crossover and mutation. Moreover, it is convenient to use the pattern theorem for theoretical analysis; the disadvantage is that it is inconvenient for reflecting the specific knowledge of the problem sought, and due to the random nature of the genetic algorithm, the local search ability is poor. Many scholars have made various improvements to the coding methods of genetic algorithms. For example, in order to improve the local search ability of genetic algorithm, gray-code coding is proposed. In order to improve the computational complexity and improve the computational efficiency of genetic algorithm, floating point or integer coding is proposed. In order to facilitate the use of problem-solving expertise and to promote the mixed use of related approximation algorithms, a symbol encoding method is proposed. The purpose of image correlation matching is to find the best matching position of the template whose coordinates are the optimal solution for image correlation matching. In this paper, considering the particularity of image correlation matching and using integer coding, each chromosome contains two genes, horizontal and vertical coordinate values. For example, chromosome A is Ca(*x*, *y*). In the genetic algorithm processing flow, the coded design task is the initial population setting, until the evolution from one generation to another ceases” according to some evolution termination criteria. The most common initial method is undirected random initialization. Instead of using the traditional method of randomly generating the initial population, this paper adopts the sampling method, that is, extracts several points on the image as the initial population at regular intervals. For example, if the size of the image to be matched is 256 × 256 and the initial overall setting is 100, a 10 × 10 grid is superimposed on the image to be matched. All intersections can be the initial population. This initialization method ensures that the initialized individuals are evenly distributed throughout the solution space, with the best matching points being obtained with fewer individuals and iterations. The flowchart of the genetic algorithm with self-recognition ability is shown in Figure 1.

RETRACTED

In genetic algorithms, the convergence of the algorithm is directly related to the choice of crossover probability and mutation probability. The probability of crossing determines the update speed and search speed of the population. It is easy to search for new good individuals and speed up the convergence of the algorithm, but if it is too large, it is very likely to destroy the existing high performance mode of the population; if it is too small, it will make the search stagnant, and the algorithm will be in a “dull” state. The possibility of mutation is an important means of maintaining population diversity and preventing precocity. If it is too big, it will make the genetic algorithm a random search and lose its purpose. In this regard, domestic and foreign scholars have done a lot of research and proposed different adaptive methods to improve genetic effects in some aspects. However, there are still deficiencies in protecting the good individuals of the population from being destroyed, and the crossover operation of individuals with high fitness is performed with a low probability. Those with poor fitness are likely to cross. This protects the overall fitness of the population, but it hinders the creation of new and superior individuals. From the whole process of population evolution, the algorithm often has a problem of slow convergence or even small energy convergence in the late stage of operation. If the cross probability is with high probability in the early stage of evolution, the evolution cycle is constant and small. The probability value is made. Then, such problems will be effectively improved. In the evolutionary process, the genetic algorithm needs to equalize opportunities in the search optimization area so as to ensure that each individual in the population has an equal probability of crossover. This paper uses the genetic algebra of crossover and probability:

(1) $$\begin{array}{c} P_{c}=\frac{1}{1+e^{\alpha G}}+\beta , \end{array}$$

where *G* is the genetic generation, *P*_*c*_ is the curvature change, and *ß* is a convergence limit.

RETRACTED

The mutation operator is derived from the concept of mutation of the biological gene and is a supplementary method for generating new genes. At the same time, it determines the local optimization ability of the genetic algorithm. The appropriate mutation probability can ensure that the genetic algorithm does not show “premature” phenomenon. In the initial stage, the diversity of the population is relatively rich, so the mutation rate should be small so as to ensure the running speed of the algorithm. As evolution progresses, individuals tend to be more adapted to their surroundings, resulting in a reduction in individual diversity. At this time, in order to maintain the diversity of the population, the mutation rate should be larger, and for individuals with a lower mutation probability whose fitness value is higher than the average fitness of the population, in order to protect the next generation, those individuals whose fitness value is lower than the average fitness degree value, the mutation rate should be higher. Based on this, this paper designs adaptive mutation probability related to genetic algebra and individual fitness:

(2) $$\begin{array}{c} P_{m}=\left\{\begin{array}{cc} P_{m1}, & f>f_{\text{avg}},\\ \frac{e^{\gamma G}-1}{e^{\gamma G}+1}\cdot \frac{f_{\max}-f}{f_{\max}-f_{\text{avg}}}\text{,} & f\leq f_{\text{avg}}, \end{array}\right. \end{array}$$

where *G* is genetic algebra; *γ* is the rate of change or variation; *f* is the fitness value of the individual to be mutated; *f*_*avg*_ is the average fitness value of the population; and *P*_*m1*_ is a large variation of probability values, being generally 0.1.

## 3. Experiments

The genetic algorithm is improved, and the results are compared with the basic genetic algorithm analysis. Verify the operational parameter settings used by the improved genetic algorithm: population size *M* = 80; evolution algebra *T* = 200; the variable number of the binary code is 2, and the chromosome length is 40; distance between niches *L* = 0.5; function f1 is the Shubert function, a commonly used genetic algorithm test function.

RETRACTED

This function is a local optimum, of which the 18th is a global optimum.

(3) $$\begin{array}{c} \min f_{1}\left(\max\right)=\left\{\sum_{i=1}^{5}i\;\cos\left[\left(i+1\right)x+i\right]\right\}\times \left\{\sum_{i=1}^{5}i\;\cos\left[\left(i+1\right)y+i\right]\right\},-10\leq x,y\leq 10,\\ \max f_{2}\left(\max\right)=0.5-\frac{\sin^{2}\sqrt{\left(x^{2}+y^{2}\right)}-0.5}{\left[1+0.001\left(x^{2}+y^{2}\right)\right]},-100\leq x,y\leq 100. \end{array}$$

When testing the performance of NAGA, since the minimum value is obtained, the objective function value *f* (*X*) is transformed into the individual fitness F (*X*) by the following formula:

(4) $$\begin{array}{c} \text{F}\left(x_{1},x_{2}\right)=\left\{\begin{array}{cc} 1-0.05f\left(x_{1},x_{2}\right), & f\left(x_{1},x_{2}\right)<0,\\ 1, & f\left(x_{1},x_{2}\right)\geq 0. \end{array}\right. \end{array}$$

The similarity measure is a measure used to determine the similarity between features to be matched. It is usually defined as a cost function or a form of a function. In the image matching process, distance, similarity, and probability measures are the three most commonly used measures.

Set vector $\bar{x}={\left[x_{1},x_{2}\cdots x_{n}\right]}^{T}$, a sequence of features representing a template, and vector $\bar{y}={\left[y_{1},y_{2}\cdots y_{n}\right]}^{T}$. The distance measure represents the sequence of features to be matched and has the following manifestations. Mean square error of two images is as follows:

(5) $$\begin{array}{c} \bar{x}-\bar{y}={\left[y_{1}-x_{1},y_{2}-x_{2}\cdots y_{n}-x_{n}\right]}^{T}. \end{array}$$

Root mean square error is as follows:

(6) $$\begin{array}{c} S=\sqrt{{\left|y_{1}-x_{1}\right|}^{2}+{\left|y_{2}-x_{2}\right|}^{2}+\cdots +{\left|y_{n}-x_{n}\right|}^{2}}. \end{array}$$

*S* is the square root of the distance between points *x* and *y* in the *n*-dimensional space. Intuitively, the smaller the distance, the stronger the similarity.

### 3.1. Absolute Difference and Distance (Block Distance)

The difference absolute value sum is the sum of the absolute values of the differences between the vectors $\bar{x}$ and $\bar{y}$, i.e.,

(7) $$\begin{array}{c} S=\left|y_{1}-x_{1}\right|+\left|y_{2}-x_{2}\right|+\cdots +\left|y_{n}-x_{n}\right|=\sum_{i=1}^{n}\left|y_{i}-x_{i}\right|. \end{array}$$

There is also an average difference absolute value:

(8) $$\begin{array}{c} S=\frac{1}{n}\sum_{i=1}^{n}\left|y_{i}-x_{i}\right|. \end{array}$$

The Mahalanobis distance calculation formula is as follows:

(9) $$\begin{array}{c} M={\left(\bar{y}-\bar{x}\right)}^{T}\overset{-1}{\underset{y}{\sum }}\left(\bar{y}-\bar{x}\right). \end{array}$$

In the formula, $\bar{y}$ is assumed to be a normal distribution with a covariance matrix. The larger the distance on the correlation, the higher the similarity, and the smaller the distance between the components of the feature vector, conversely, the smaller the distance on the correlation, the lower the similarity, and the greater the distance between the components of the feature vector. The main frequency of the experiment is 3.6 GHz, a hardware host running environment with 6 GB memory is set up, and the experiment is carried out on the MATLAB 7.0 software platform.

RETRACTED

The parameters of the genetic algorithm in the experiment are as follows: population size *M* = 80, evolution algebra *G* = 20, crossover probability *P*_*c*_ = 0.8, and mutation probability *P*_*m*_ = 0.01. The experimental diagram is shown on the left of Figure 2 and Figure 3. For comparison with the traditional image matching algorithm, gray-scale correlation matching is used, and the similarity function adopts the average squared difference.

The POC algorithm is a nonlinear frequency domain correlation algorithm based on the Fourier power spectrum. Because this method only takes the phase information in the cross power spectrum, it reduces the dependence on the image content, and the obtained correlation peaks are sharp. Therefore, the displacement detection range is larger and the matching accuracy is high. In addition, the phase correlation technology is less dependent on the image gray level and has a certain anti-interference ability. However, it is particularly sensitive to image rotation. The RIPOC algorithm can make up for its shortcomings. The rotation-invariant phase correlation method can judge whether two images with rotation are related or not and can measure the rotation angle of the two images without considering the position of the rotation axis.

The similar data detection algorithm calculates the similarity ([0, 1]; 1 means identical) or distance ([0, 1]; 0 means identical) for a given pair of data sequences to measure the similarity between the data. Based on the algorithm of multiresolution tower structure, the two core issues of learning model design and matching algorithm are mainly studied. The established image pyramid has the disadvantage of insufficient high-frequency details for extraction. The multiresolution tower fusion algorithm is applied to the establishment of the Laplacian pyramid, and the obtained learning model can be more abundant and effective in multiscale and multiresolution training. In addition, a new idea is introduced in the matching restoration process. First, search for the 4 most matching high-frequency details in the Laplacian pyramid, and then use the weighted average of these 4 high-frequency details as the height of the missing face image. Compared with the method of using a single best matching high-resolution block for restoration, this method can obtain more complete high-frequency information.

RETRACTED

## 4. Discussion

Experiments were performed in MATLAB. The results of arithmetic operation described herein with new adaptive genetic algorithm (AGA) are compared. The definition of the correct matching precision = number of matches/experimental times × 100%. The comparison of the experimental data is shown in Table 1.

Compared with the other two matching algorithms, this paper has a significant improvement in performance, as shown in Table 2.

The left halves of Figures 2 and 3 of 900 × 600 are the images to be matched. From the baseline implementations of 2 and 3, the top 100 are the most confident feature matches. In this case, 93 are correct (highlighted in green) and 7 are incorrect (highlighted in red).

The experimental results of the images to be matched show that the proposed algorithm can achieve accurate matching in a short time, with better speed than the traditional AGA algorithm. At all matching positions, the matching result is the same as the traditional method. The SSDA algorithm is about twice as fast as the original algorithm in the matching calculation, but the required calculation time and the position of the matching template in the image have very large relationship. For the same matching effect, the speed of the genetic algorithm is more than an order of magnitude higher than that of the SSDA algorithm, and the matching time is basically constant (the calculation amount fluctuation caused by the random decision operation in the genetic algorithm can be ignored). It can be seen from Figure 4 that the optimal horizontal position converges to 70 after 500 generations of inheritance, and the vertical position converges to the ideal position after 350 generations. The algorithm is stable and precisely matches the ideal position.

## 5. Conclusion

Genetic algorithm is a random search optimization process. It greatly reduces the search space, greatly reduces the amount of calculation, and improves the optimization efficiency. Because the algorithm is simple, easy to understand, easy to operate, and simplifies complex problems, it is becoming more and more popular. Based on the collection and review of a large body of domestic and foreign literature, this paper summarizes and analyzes the research results of predecessors. First, the development, basic principles, structure, and application of genetic algorithms are introduced. An improved genetic algorithm is proposed. Second, the basic ideas and research status of image matching are studied and discussed. However, the matching efficiency has not reached people's ideal state, and the application of genetic algorithm greatly improves the matching efficiency. In this paper, the traditional genetic algorithm is used to solve the problem that the optimization problem has slow convergence and low maturity. A crossover operator with self-recognition capability is used to maintain population diversity when performing cross-operations. The experimental results show that, compared with the traditional genetic algorithm, the improved genetic algorithm has achieved good results in terms of algorithm fastness and matching accuracy. It can be used for image template matching with higher real-time performance, that is, the research on the identification and tracking of dynamic targets.

RETRACTED

## Figures and Tables

**Figure 1:** Algorithm flowchart.

**Figure 2:** Positive feature matching.

**Figure 3:** Side feature matching.

**Figure 4:** Fitness function curve.

**Table 1:** Performance comparison between AGA population size and algorithm population size.

Algorithm	Matching precision (%)	Average running time (s)
AGA population size	*N* = 50 57	3.1635
	*N* = 100 77	5.5870
	*N* = 150 77	8.7488
	*N* = 200 90	11.4235

Algorithm population size	*N* = 50 42	2.0110
	*N* = 100 58	2.5834
	*N* = 150 91	3.2170
	*N* = 200 100	5.3217

**Table 2:** Performance comparison table.

Matching algorithm	FPGA	Speed (ms)
A	EP2S90F78014	118.7
B	EP3SL340F1517C3	53.6
This article	XC2VP30	31.71

## Data Availability

This article does not cover data research. No data were used to support this study.
